This article has been retracted.

# Effects of Neonatal Feeding Patterns on Infant Health

**DOI:** 10.1155/2022/2225415

**Published:** 2022-02-15

**Authors:** Shi Xiaoli, Hao Weiyan, Dandan Li

**Affiliations:** ^1^Neonatal Care Unit of Pediatric Internal Medicine, Laizhou People's Hospital, Yantai, 261400 Shandong, China; ^2^Pharmaceutical Engineering, Pharmaceutical Engineering Part, Jiangsu Ocean University, 222005 Lianyungang, Jiangsu, China

## Abstract

**Objective:**

Early and reasonable feeding mode can not only ensure the good nutritional condition of infants but also enhance the infant immunity and resistance, which has a certain role in promoting health and preventing the occurrence of chronic diseases in adulthood. In this study, the effect of neonatal feeding methods on the infant body, the influence of early feeding on the growth rate, and development of infants aged 0-3.

**Method:**

From January 2016 to June 2019, a total of 600 infants who have been systematically managed in our hospital since birth were selected. All newborns were 37-40 weeks old, weighing 2350-4100 g, without congenital diseases. They were grouped according to feeding methods. 194 infants were exclusively breastfed, 32.3%; 207 people were artificially fed, 34.5%; 199 people were mixed fed, 33.2%. The Kaup index method was used to judge the nutritional status. Developmental Screening Test for ages 0 to 6 (DST) and Bailey Infant Development Scale (BIDS) were used to rate the intellectual and behavioral development of infants and children. According to the growth and development reference standard of 0 ~ 4-year-old children recommended by who in 2006, the age weight standard deviation score (WAZ), age length (height) standard deviation score (HAZ), and body (long) height-weight standard deviation score (WHZ) were performed, and the statistical analysis was performed with SPSS24.0 software. The height, weight, intelligence, and motor development of infants in the three groups at 1 month, 3 months, 6 months, 12 months, 24 months, and 36 months were analyzed and compared, and the test results were recorded in detail.

**Result:**

There was no significant difference in 3-month-old WAZ and HAZ among the three groups (*P* > 0.05). Within 6 months, the WAZ and HAZ values of the pure breastfeeding group and mixed feeding group were higher than those of the artificial feeding group (*P* < 0.05). From 6 months to 12 months, the WAZ and HAZ values of the artificial feeding group were better than those of artificial feeding group and mixed feeding group (*P* < 0.05). The scores of MI, DQ, PDI, and MDI in the mixed feeding group within 12-36 months were slightly higher than those in the breastfeeding group and significantly better than those in the artificial feeding group (*P* < 0.05). The prevalence of the breastfeeding group was 22.2% (43/194) and mixed feeding group was 19.8% (39/199), which was lower than that of the artificial feeding group 57.8% (120/207), *P* < 0.01. The number of people with normal psychological development was 88.7% (172/194) in the breastfeeding group and 88.9% (177/199) in the mixed feeding group, which was higher than 76.3% (158/207) in the artificial feeding group (*P* < 0.01).

**Conclusion:**

When there is little colostrum secretion in the first 2-3 days of delivery, appropriate addition of formula milk can reduce the incidence of diseases in newborn infants. Breast milk is the most perfect natural food. The immune substance in breast milk is an important element for infants to resist diseases. The communication between mother and child is the first condition for the development of infant mental health.

## 1. Introduction

The growth and development of 0-3-year-old infants will determine their life-long health. If they are malnourished at this stage, it will affect their future growth and development and will also have a certain impact on their intellectual development. The neonatal period is the most important period in one's life. Therefore, the early reasonable feeding mode can not only ensure the good nutritional status of infants but also enhance the immunity and resistance of infants, which plays a certain role in promoting health and preventing the occurrence of chronic diseases in adulthood [1].

Early infant feeding methods include breastfeeding, mixed feeding, and artificial feeding. In breastfeeding, there is breastfeeding only, no other liquids. In mixed feeding, in the early stage of parturient women, in addition to breast milk, we increase the milk adding device next to the milk to add formula milk according to whether the baby cries, looks for food, and the number of urination of the baby every day. After the parturient women lactate, they will give all breast milk and feed the baby with water or fruit juice. In artificial feeding, breastfeeding is not possible for various reasons, and only formula milk is used. In 2016-2020, institutions studied the impact of different feeding methods on infant developmental behavior and found that there are great differences in the development behavior and nutritional status between artificial feeding and breastfeeding [2]. At present, there are many comparative investigation reports on artificial feeding and breastfeeding, but there are few investigations on the relationship between mixed feeding, breastfeeding, and artificial feeding.

In order to explore the influence of different ways of early feeding methods on growth rate, growth level, and physical development of 0-3-year-old infants, this study was conducted through the feeding method of 600 infants born from January 2019 to June 2019; systematically managed by our hospital, the height, weight, intelligence, and exercise level of infants were tested in a month, and the test results were recorded in detail. In investigation and analysis by using a bivariate *t*-calibration, the aim is to provide reference materials for guiding reasonable feeding and improving the intelligence and behavioral development of infants and young children.

## 2. Data and Methods

### 2.1. Infant Data

We study 600 newborns born in our hospital from January 2019 to June 2019, with a gestational period of 37-40 weeks, a weight of 2350-4100 g, and no congenital diseases (see Figure 1 for details).

Among them, there were 321 male infants, accounting for 53.5%, and 279 female infants, accounting for 46.5%. According to the feeding methods, 194 people were exclusively breastfed, accounting for 32.3%; 207 people were artificially fed, accounting for 34.5%; 199 people were mixed fed, accounting for 33.2%. The height, weight, intelligence, and motor development of infants were measured in month, and the test results were recorded in detail.

### 2.2. Physical Indicators

We use the same instrument to measure the weight and height of infants. The nutritional status was determined by the Kaup index method. The Kaup index is also known as the body mass index, proposed by Kaup in 1921, modified by Davenport etc.; therefore, it is also called the Kaup-Davenport index. It refers to the number of body weight contained in the unit area, so it is closely related to the sebum thickness, and it is a better measure of nutritional status and obesity [3]. Kaup index = [weight (kg)/height (cm)^2^] × 104. Kaup index < 15 is lean, 15-19 is normal, 19-22 is excellent and tends to be overweight; and >22 is obese [4]. According to the growth and development reference standard of 0 ~ 4-year-old children recommended by WHO in 2006, age-specific weight standard deviation score (WAZ), age-specific body length (height) standard deviation score (HAZ), and body length (height) height-weight standard deviation score (WHZ) [5]. The intelligence and behavioral development of infants and young children were assessed by the development screening test for 0 ~ 6 years (DST) and Bailey infant development scale (BSID) [6]. DST mainly measured the following four abilities: human ability (children's ability to respond to people around them and take care of their own life), material ability (children's ability to see, pick things and draw pictures by hand), speech ability (infant's ability to listen and understand language), and rough motor ability (infant's ability to sit, walk and jump). Intellectual development is evaluated by development quotient (DQ): DQ < 70 is abnormal, 70-84 is suspicious, and ≥85 is normal; motor development index (MI) is used to evaluate infant's motor development [7]. BSID is evaluated by the intellectual development index (MDI) and psychomotor development index (PDI). To evaluate the intelligence and action development of infants, the total score is 100. The score were positively associated with intellectual and behavioral development in infants and young children [8].

### 2.3. Feeding Method

We judge by the feeding mode 6 months after birth: (1) breastfeeding, only breastfeeding without other liquids; (2) mixed feeding: in the early stage of parturient women, in addition to breast milk, we increase the milk adding device next to the milk to add formula milk according to whether the baby cries, looks for food, and the number of urination of the baby every day. After the parturient women lactate, they will give all breast milk and feed the baby with water or fruit juice. (3) Artificial feeding: breastfeeding is not possible for various reasons, and only formula milk is used.

### 2.4. Statistical Methods

All arithmetic mean values and standard deviation rates are statistically expressed in ($\bar{x}\pm s$), t calibration. The counting data are expressed in (%), chi-square test and analysis of variance are used according to the nature of the data, and the data are analyzed by SPSS 24.0 statistical analysis software.

The *t* value and *P* value of bivariate *t*-check come from the bivariate *t*-check process, where the *t* value is the value of the output result. When *t* > 10.000, the two columns of data were considered to have a large proportion of credible statistical differences, and the greater the *t* value, the greater the statistical difference; the *P* value is the log value of the output result. When *P* < 0.05, it is considered that the result data is within the confidence space. When *P* < 0.01, it is considered that the result data has significant statistical significance. The smaller the *P* value, the higher the degree of confidence. Subjected to the length, only the calculation algorithm of the *t* value (value) is explained here, such as

(1) $$\begin{array}{c} t_{\text{Value}}=\frac{\bar{x}-\mu }{S/\sqrt{n-1}}, \end{array}$$

where $\bar{x}$ is the arithmetic mean of the investigated sample sequence, *μ* is the average value of the reference sample sequence, *n* is the number of nodes of the investigated sample sequence, *m* is the number of nodes in the reference sample sequence, and *S* is the standard deviation rate of the investigated sample sequence.

The arithmetic mean value in formula (1) is shown in

(2) $$\begin{array}{c} \bar{x}=\frac{1}{n}\overset{n}{\underset{i=1}{\sum }}x_{i},\\ \mu =\frac{1}{m}\overset{m}{\underset{i=1}{\sum }}x_{i}, \end{array}$$

where *i* is the traversal pointer, *M* is the number of nodes of the reference sample sequence, and *x*_*i*_ is the *i*th input value in the sequence. The meaning of mathematical symbols is the same as above.

The algorithm of standard deviation rate in formula (1) is shown in

(3) $$\begin{array}{c} S=\frac{1}{n-1}\sqrt{\overset{n}{\underset{i=1}{\sum }}{\left(x_{i}-\bar{x}\right)}^{2}}. \end{array}$$

## 3. Results

### 3.1. Analysis of Physical Development of Three Groups at Different Months

See Table 1 for details of physical development of infants of different months under different feeding methods.

There was no significant effect of different feeding methods on the height in the three groups within 3 months (*t* = 23.068, *P* > 0.05). Within 3-6 months, the artificial feeding group was lower than the other two groups, *t* = 9.953, *P* < 0.05, with a credible statistical difference. At 6-12 months, the artificial feeding group was higher than the other two groups, *t* = 9.782, *P* < 0.05. The height data of newborns in the breastfeeding group and mixed feeding group were statistically consistent, *t* = 46.832, *P* > 0.05. The height data were observed for 36 months. It was found that there was no statistical difference in other time periods except the above 3 ~ 6 months, and the results were credible, *t* > 10.000, *P* < 0.05.

See Table 2 for details of weight analysis of infants of different months under different feeding methods.

In the results of weight comparison in Figure 2, the weight development of the artificial feeding group was higher than that of the other two groups, with a large proportion of credible statistical difference. Within 3-6 months, the weight development of newborns in the artificial feeding group was relatively slow, *t* = 7.172, *P* < 0.05, with significant statistical difference. Between 6 months and 12 months, the weight development rate of the artificial feeding group increased and gradually exceeded that of the breastfeeding group and the mixed feeding group. At this time, *t* = 6.265 and *P* < 0.05, there was a credible statistical difference. After 12 months, the development speed of the artificial feeding group was further accelerated and the gap between the artificial feeding group and the other two groups was widened. At this time, *t* = 3.879 and *P* < 0.05, with a large proportion of credible statistical difference, there was a credible statistical consistency between the weight data of the breastfeeding group and mixed feeding group, *t* > 10.000, *P* < 0.05.

See Table 3 for details of the Kaup index analysis of infants of different months under different feeding methods:

There was no significant difference in 3-month-old WAZ and HAZ among the three groups (*t* = 31.215, *P* > 0.05). Within 6 months, the WAZ and WHZ values of the artificial feeding group were lower than those of the other two groups, *t* = 5249, *P* < 0.05. From 6 months to 12 months, the WAZ and WHZ values in the artificial feeding group were higher than those in the other two groups (*P* < 0.05). Within 12-36 months, the WHZ value of the artificial feeding group was significantly higher than that of the other two groups, and the incidence of obesity was higher than that of the other two groups. Compared with the other two groups, the artificially fed children had an increased risk of overweight and obesity.

It can be seen from Table 2 and Figures 3 and 4 that the lean rate and obesity rate of artificial feeding are higher than those of breastfeeding and mixed feeding. There is little difference between breastfeeding and mixed feeding.

### 3.2. Analysis of DST and BSID Test Results of Infants with Different Feeding Methods

See Table 4 for details of DST and BSID test results of infants of different months under different feeding methods:

Among the 600 infants surveyed, in the scores of MI, DQ, PDI, and MDI, there was a small credible difference between the mixed feeding group and the breastfeeding group, which was higher than that in the artificial feeding group, with a large proportion of credible statistical difference, *t* = 3.262, *P* < 0.05.

### 3.3. Effects of Different Feeding Methods on Physical and Mental Health of Infants

See Figure 5 for details of physical health of infants of different months under different feeding methods.

In Figures 5 and 6, within 36 months, the prevalence of infants and young children was 22.2% (43/194) in the breastfeeding group and 19.8% (39/199) in the mixed feeding group, which was lower than 57.8% (120/207) in the artificial feeding group (*t* = 8.055, *P* < 0.01); the number of infants and young children with normal psychological development was 88.7% (172/194) in the breastfeeding group and 88.9% (177/199) in the mixed feeding group, which was higher than 76.3% (158/207) in the artificial feeding group (*t* = 2.990, *P* < 0.01).

## 4. Discussion

Infants are the key period of children's growth and development, and the choice of the feeding mode is directly related to the physical development of infants in the future. In this study, participants were tracked to 3 years old and measured in different periods. The results showed that (1) different feeding methods had no significant effect on the height of infants. There was no significant effect of different feeding methods on height in the three groups within 3 months (*t* = 23.068, *P* > 0.05). Within 3-6 months, the artificial feeding group was lower than the other two groups, *t* = 9.953, *P* < 0.05, with a credible statistical difference. At 6-12 months, the artificial feeding group was higher than the other two groups, *t* = 9.782, *P* < 0.05. The height data of newborns in the breastfeeding group and mixed feeding group were statistically consistent, *t* = 46.832, *P* > 0.05. The height data were observed for 36 months. It was found that there was no statistical difference in other time periods except the above 3 ~ 6 months, and the results were credible, *t* > 10.000, *P* < 0.05. (2) In the results of weight comparison, the weight development of the artificial feeding group was higher than that of the other two groups, with a large proportion of credible statistical difference. Within 3-6 months, the weight development of newborns in the artificial feeding group was relatively slow, *t* = 7.172, *P* < 0.05, with significant statistical difference. Between 6 months and 12 months, the weight development rate of the artificial feeding group increased and gradually exceeded that of the breastfeeding group and the mixed feeding group. At this time, *t* = 6.265 and *P* < 0.05, there was a credible statistical difference. After 12 months, the development speed of the artificial feeding group was further accelerated and the gap between the artificial feeding group and the other two groups was widened. At this time, *t* = 3.879 and *P* < 0.05, with a large proportion of credible statistical difference, there was a credible statistical consistency between the weight data of the breastfeeding group and mixed feeding group, *t* > 10.000, *P* < 0.05. (3) Compared with mixed feeding and breastfeeding, artificially fed children have an increased risk of overweight and obesity. There was no significant difference in 3-month-old WAZ and HAZ among the three groups (*t* = 31.215, *P* > 0.05). Within 6 months, the WAZ and WHZ values of the artificial feeding group were lower than those of the other two groups, *t* = 5249, *P* < 0.05. From 6 months to 12 months, the WAZ and WHZ values in the artificial feeding group were higher than those in the other two groups (*P* < 0.05). Within 12-36 months, the WHZ value of the artificial feeding group was significantly higher than that of the other two groups, and the incidence of obesity was higher than that of the other two groups. Compared with the other two groups, the artificially fed children had an increased risk of overweight and obesity [9]. (4) In the scores of MI, DQ, PDI, and MDI, there was a small credible difference between the mixed feeding group and the breastfeeding group, which was higher than that in the artificial feeding group, with a large proportion of credible statistical difference, *t* = 3.262, *P* < 0.05. (5) The prevalence of infants and young children within 3 years are as follows: 22.2% (43/194) in the breastfeeding group, 19.8% (39/199) in the mixed feeding group, lower than 57.8% (120/207) in the artificial feeding group (*t* = 8.055, *P* < 0.01); the number of infants and young children with normal psychological development are as follows: 88.7% (172/194) in the breastfeeding group, 88.9% (177/199) in the mixed feeding group, and higher than 76.3% (158/207) in the artificial feeding group (*t* = 2.990, *P* < 0.01).

During this time, many studies have found that in modern years, in recent years, a large number of studies have found that breast milk contains substances that promote the development of infant brain cells. Breast milk contains long-chain polyunsaturated fatty acids DHA and AA necessary for brain development, which can promote brain cell development and lay a material foundation for improving infant MDI and PDI, especially for infants under 6 months old [10]. However, the content of these substances in traditional formula milk is very small and almost negligible [11]. It has been found that the concentration of sialic acid (SA) in the frontal cortex of breast-fed infants is higher than that of artificially fed infants. This may promote the formation of synapses, help infants form a more stable structural basis for memory, and strengthen the development of the nervous system. The content of sialic acid in formula is significantly lower than that in breast milk [12]. Breast milk also contains more taurine, which is 10~30 times that of cow's milk. Taurine is a nerve growth regulator and can promote infant brain development. In addition to the great benefits of breast milk itself to the brain development of infants, the process of breastfeeding is also conducive to the neural development of infants [13].

Breast milk is an ideal food for the healthy growth and development of infants. Immunoglobulin in breast milk is an important element for infants to resist diseases, it can improve immunity, intelligence, and mother-child feelings for infants. Sufficient milk is an important prerequisite for the success of breastfeeding [14]. However, the colostrum secretion of the parturient is very small 2-3 days after delivery, and some infants are in a state of hunger. The appropriate addition of formula milk can reduce the disease of newborn infants. The occurrence of neonatal jaundice is related to the insufficient amount of early breast milk and insufficient water supplement. In addition, it can also avoid the impact on the brain development of newborns due to insufficient protein [15]. Before enough milk comes out, blindly let the baby suck more, which will affect the baby's sleep and affect the development of the baby's central nervous system [16].

The data of this paper show that mixed feeding in the early stage of birth can not only provide rich nutrition for infants but also do not affect the all-round development of infants. It is superior to artificial feeding and breastfeeding in terms of intelligence and physical development of infants. Mixed feeding is a combination of the advantages of breastfeeding and artificial feeding. It can make up for the defects in the early stage of exclusive breastfeeding, reduce the excessive dependence of infants on breast milk, and delay the addition of complementary foods.

The outcome of this study is accordant with the previous studies, which further confirmed that the mixed feeding mode of breast milk and formula milk has advantages in ensuring the healthy growth of newborns and young children.

## 5. Summary

The results of this study are consistent with the results of the above scholars, which further confirms that the mixed feeding mode based on breast milk and supplemented with formula has higher advantages in ensuring the normal growth and development of infants and young children. However, this study did not investigate and analyze the supplementary food addition. The time domain of infant observation is still short, so it is not possible to further analyze the impact of different feeding methods on children. The results still need to be confirmed in the future data collection.

## Figures and Tables

**Figure 1:** Analysis of basic data of infants and young children.

**Figure 2:** Effects of feeding methods in different periods on weight development.

**Figure 3:** Trend of lean rate in different feeding methods.

**Figure 4:** Trend of obesity rate in different feeding methods.

**Figure 5:** Comparison of infant diseases.

**Figure 6:** Comparison of infants with normal psychological development.

**Table 1:** Effects of feeding methods in different periods on height development ($\bar{x}\pm$s, cm).

Feeding mode	Breastfeeding	Artificial feeding	Mixed feeding
1 m	55.2 ± 2.1	55.1 ± 2.3	55.3 ± 2.2
3 m	62.5 ± 3.4	63.4 ± 2.9	62.7 ± 3.3
6 m	72.9 ± 3.6	68.3 ± 3.2	73.2 ± 3.5
12 m	76.9 ± 3.4	78.9 ± 3.8	77.1 ± 3.2
24 m	88.7 ± 2.6	89.6 ± 2.5	89.2 ± 3.0
36 m	98.6 ± 3.3	99.6 ± 3.2	98.8 ± 3.6

**Table 2:** Effects of feeding methods in different periods on body weight development ($\bar{x}\pm$s, kg).

Feeding mode	Breastfeeding	Artificial feeding	Mixed feeding
1 m	4.80 ± 0.66	4.75 ± 0.50	4.81 ± 0.65
3 m	6.78 ± 1.55	6.35 ± 1.64	6.80 ± 1.58
6 m	8.43 ± 0.95	8.59 ± 1.36	8.44 ± 0.99
12 m	10.24 ± 1.12	10.77 ± 1.43	10.36 ± 1.19
24 m	12.77 ± 1.32	13.38 ± 1.43	12.81 ± 1.34
36 m	15.25 ± 1.45	16.11 ± 1.88	15.28 ± 1.47

**Table 3:** The Kaup index under different feeding methods.

Feeding mode	Kaup	1 m	3 m	6 m	12 m	24 m	36 m
Breastfeeding	<15	7	6	8	10	11	10
	15-22	171	158	158	165	167	175
	>22	16	30	28	19	16	9

Artificial feeding	<15	33	31	23	18	19	12
	15-22	151	148	144	155	152	169
	>22	13	28	40	34	36	28

Mixed feeding	<15	9	8	6	7	8	9
	15-22	175	167	168	171	173	178
	>22	15	24	25	21	18	12

*t*		-2.152	-2.366	-0.006	-0.751	-1.507	-2.044

*P*		0.032	0.031	0.997	0.453	0.131	0.042

**Table 4:** Analysis of DST and BSID test results of infants with different feeding methods.

Feeding mode	MI	DQ	PDI	MDI
Breastfeeding	98.89 ± 10.82	98.45 ± 10.59	102.58 ± 8.72	102.82 ± 9.41
Artificial feeding	85.34 ± 10.45	84.21 ± 12.66	85.45 ± 8.43	84.72 ± 7.66
Mixed feeding	99.68 ± 10.83	98.51 ± 10.62	103.02 ± 8.73	102.84 ± 9.43

## Data Availability

The data underlying the results presented in the study are available within the manuscript.
